# Study on the Predictive Value of P53 Protein Expression in Brain Metastasis in NSCLC and the Mechanism of miR-424 Reversing Platinum Resistance in NSCLC

This article has been retracted.

**DOI:** 10.1155/2022/5273772

**Published:** 2022-08-08

**Authors:** Yan Deng, Zhiwen Duan, Jie Luo, Wen Deng, Rongqing Liao

**Affiliations:** ^1^Department of Radiotherapy, First Affiliated Hosppital of Kunming Medical University, Kunming 650032, China; ^2^Department of Infectious Disease, First Affiliated Hosppital of Kunming Medical University, Kunming 650032, China

## Abstract

In order to analyze the predictive value of P53 protein expression in brain metastases in NSCLC and the mechanism of miR-424 reversing platinum resistance in NSCLC, a retrospective analysis is conducted in this study. Eighty-two NSCLC patients who received relevant diagnosis and treatment in our hospital from September 2020 to September 2021 are chosen. The prognosis of the patients is observed, and the patients were divided into two groups according to the occurrence of BMS. The comparison of clinical baseline data and the expression of P53 protein and miR-424 after surgery are performed. Furthermore, the predictive value of the P53 protein gene on the occurrence of BMS in NSCLC is analyzed by the ROC curve, and the expression of miR-424 in serum of the patients before and after drug resistance is compared. The results demonstrate that the expression of P53 protein has a high predictive value for predicting the occurrence of BRAIN metastases in NSCLC patients. Also, the high expression of miR-424 suggests that it is closely related to the occurrence of platinum resistance in NSCLC patients.

## 1. Introduction

Lung cancer is a common malignant tumor that occurs in the lungs of patients in clinical practice. Relevant clinical research data show that the number of lung cancer patients in China is increasing year by year, and the five-year survival rate of patients is less than 20% [1]. At present, non-small-cell lung cancer (NSCLC) still lacks sensitive and effective diagnostic markers. This is also one of the main reasons for the high mortality of NSCLC patients [2]. At present, most patients with non-small-cell lung cancer are treated by conventional radiotherapy, stereotactic radiotherapy for brain metastases, and surgical resection of brain metastases. However, the expected effect is not ideal, which easily leads to a poor prognosis. Therefore, it is necessary to identify effective clinical diagnostic markers. In addition, optimizing and improving the clinical diagnosis and treatment plan are of great significance to improve the prognosis and survival rate of patients with non-small-cell lung cancer, and it is also an important issue to be solved urgently in the current medical field [3, 4].

At present, scholars in the medical field have found that P53 protein is a very important tumor suppressor gene through studies. P53 is a tumor suppressor gene in the human body, which can be divided into wild type and mutant type [5]. Wild type is a normal gene, while mutant type is caused by mutation of a wild-type gene, which may induce other diseases. The P53 gene can kill cancer cells, and a positive test often indicates that patients may have cancer [6]. However, P53 not only kills cancer cells but also repairs damaged cells. Therefore, some cancer cells damaged by chemotherapy may be restored by this gene. P53 plays a complex role in cell cycle arrest, apoptosis, and aging, all of which may help protect the genome from cumulative mutations and the transmission of these mutations to daughter cells. P53 also plays an important role in maintaining the genomic stability of pluripotent stem cells by coordinating DNA damage response and pluripotency. As a transcription factor, P53 directly activates the transcription of a large group of genes, including CDKN1A, MDM2, PERP, PMAIP1, BBC3/PUMA, and CCNG1. Also, it can directly inhibit the expression of some genes, such as MAP4 and NANOGG [7]. These P53 target genes need to mediate various P53-dependent functions in the process of maintaining genome stability [8].

Some studies have pointed out that about 1/3 of lung cancer patients have P53 gene mutation, suggesting a close relationship between P53 protein expression and the formation, occurrence, and development of NSCLC [9]. MicroRNAs (miRNAs) are a group of noncoding RNAs with 22 nt nucleotide length in cells that regulate the expression of posttranscriptional genes [10]. It has been reported that miR-424 is abnormally expressed in a variety of tumors, which is believed to be associated with the occurrence and development of malignant tumors [11]. A study on oral cancer found that miR-424 is highly expressed in oral squamous cell carcinoma and promotes the proliferation and metastasis of oral squamous cell carcinoma by regulating the SOCS2/STAT5 signaling pathway [12]. However, there are few studies on the mechanism of action and platinum resistance of miR-424 in NSCLC. Aiming to explore the expression of P53 protein in the tissues of NSCLC patients, the clinical data differences of patients with different prognoses should be analyzed. In this study, the impact of miR-424 on platinum resistance in NSCLC patients is investigated, and the results can provide more scientific data support for the diagnosis and treatment of non-small-cell lung cancer.

This paper is organized as follows: Section 2 discusses the related work, followed by the data and methods in Section 3. In Section 4, the results and analysis are proposed. Finally, in Section 5, some concluding remarks are made.

## 2. Related Work

In recent years, with the development of science and technology, medical devices, and various new drugs, the treatment of NSCLC has been optimized to a certain extent [13]. It should be noted that the human body environment is complex and diverse, and the clinical symptoms and disease progression of different NSCLC patients are personalized. A variety of factors and molecular mechanisms in patients have an impact on the therapeutic effect of adjuvant chemotherapy [10]. Clinically, most patients with bladder cancer in postoperative therapy and chemotherapy after the illness are eased or cured, but there are still some patients at risk of tumor recurrence, progression, and metastasis, which poses a great threat to the patient's life and health, but the specific molecular mechanism is not fully proved, and it also becomes an important lesson that clinical research should focus on and pay attention to [14].

Wild-type P53 is a classic tumor suppressor gene. Clinical studies have found that P53 protein content is closely related to the stability of the body genome, cell activity, and gene repair and also plays a very important role in inducing the death of cells with difficult repair mutations [15]. Other scholars have found that the mutant P53 protein gene plays an important role in the occurrence and development of human tumors. The probability of P53 gene mutation in NSCLC is about 30%, and the stability of mutant P53 protein is significantly increased. Meanwhile, it can also form polymers with wild-type P53 protein and accumulate in the nucleus. As a result, wild-type P53 loses its tumor suppressive function, and its half-life increases, which can be detected by immunohistochemistry, so the prognosis of patients can be predicted by detecting the P53 protein expression level [16]. The results showed that the expression of P53 protein in NSCLC patients with BMS was significantly higher than that in NSCLC patients without BMS, and the analysis of P53 protein by the ROC curve had higher predictive value for the occurrence of BMS in NSCLC patients, confirming the high efficacy of P53 protein expression in predicting the prognosis of patients. The results were consistent with previous clinical studies.

At present, a number of studies have shown that miRNA is related to chemotherapy resistance of bladder cancer, and cisplatin is still the basis of chemotherapy in NSCLC in clinical practice. Therefore, some studies on miRNA related to chemotherapy resistance of NSCLC also mainly focus on cisplatin resistance. At present, several Cisplatin-related miRNAs and their intrinsic mechanisms have been successively discovered and proved [17]. miR-424 is differentially expressed in MDR-TB patients and their serum, which can be used as a biomarker for the diagnosis of MDR-TB. However, its role in tumor cell drug resistance has not been reported [18, 19]. This study conducted a follow-up investigation on the clinical efficacy of all NSCLC patients during postoperative treatment and compared the expression of miR-424 in patients in objective remission and PD patients, indicating that the relative expression of miR-424 in PD patients was lower.

## 3. Data and Methods

### 3.1. General Information

A total of 82 NSCLC patients receiving relevant diagnosis and treatment in our hospital from September 2020 to September 2021 were retrospectively analyzed, including 47 male patients and 35 female patients. Their ages range from 43 to 72, and average age is about (55.89 ± 7.75) years. The disease types of patients were adenocarcinoma (43 cases) and squamous cell carcinoma (39 cases). Clinicopathological staging is as follows: 26 stage I patients, 35 stage II patients, and 21 stage III patients.

The inclusion criteria are as follows: (1) the patients did not receive other related neoadjuvant chemotherapy before admission; (2) all patients underwent lobectomy and systematic lymph node dissection; (3) measurable lesions were found in the lungs; (4) complete clinical and pathological data; and (5) the patient has high clinical compliance and can cooperate with the relevant investigation work of this study until the end of the study.

The exclusion criteria are as follows: (1) postoperative survival time <1 month; (2) the patients did not receive standard treatment after operation; (3) patients with other malignant tumors; (4) patients with mental or consciousness disorders.

All patients in this study received adjuvant chemotherapy after surgery, and the chemotherapy regimen was EGFR-TKIs (gefitinib, erlotinib, ectinib). All patients accepted and cooperated with the relevant follow-up work of this study and were grouped according to the relevant diagnosis results such as regular postoperative review. Among them, NSCLC patients with BMS were included in the NSCLC BMS group (*n* = 34), and patients without BMS were included in the NSCLC nonmetastasis group (*n* = 48).

### 3.2. Detection Method for P53 Protein

Lung cancer tissue samples were collected from all patients after the operation. The cancer tissues and adjacent tissues were fixed with paraformaldehyde solution and paraffin-sectioned and stained with routine HE staining. The tumor cells stained with the P53 cytoplasm and nucleus were P53-positive cells. The percentage of P53-positive cells in the total number of tumor cells in the whole section was calculated by the positive rate of P53 protein expression. All the results were double-blind interpreted by two pathologists, and the positive expression rate was 1%.

### 3.3. miR-424 Detection Method

The EDTA anticoagulant tube was used to collect 6 mL fasting venous blood samples before and after drug resistance of EGFR-TKIs, and all blood samples were centrifuged. Centrifuge parameters were set at 3500 r/min, centrifuge radius was set at 10 cm, and the centrifugation lasted for 15 min. After that, the supernatant was taken and stored at −80°C for testing. Finally, the detection of miR-424 was carried out intensively, and all the kits used in the detection process were strictly operated according to the relevant instructions. Blood samples were taken from all patients after they signed informed consent.

### 3.4. Follow-Up Work

All patients underwent imaging examination at the beginning of egFR-Tkis treatment as the first assessment, and serum samples before EGFR-TKIs treatment or within 1 month of taking drugs were taken as the predrug resistance group. Then, each case was followed up regularly, with the first follow-up at the end of the first month after treatment and once every 3 months thereafter. Detailed physical examination was performed each time, and lung enhancement CT, skull plain CT, abdominal color ultrasound, and tumor markers were reviewed. In the follow-up observation, once disease progression was found in imaging assessment, EGFR-TKIs resistance was considered, and serum samples were collected as the postresistance group.

### 3.5. Observation Indicators

The details of the observation indicators are as follows: (1) comparison of baseline data; (2) the expression of P53 protein and Mir-424 was compared; (3) the ROC curve was used to analyze the predictive value of the P53 protein gene for brain metastasis in NSCLC; and (4) the expression of miR-424 in serum of patients before and after drug resistance was compared.

### 3.6. Evaluation Criteria

The clinical treatment effect of all patients in this study was evaluated according to the relevant content of the latest clinical efficacy evaluation criteria for solid tumor, which was divided into complete remission (CR), partial remission (PR), stable disease (SD), and progression disease (PD) [20, 21]. The objective effective rate is defined as (CR + PR)/(CR + PR + SD + PD) × 100%, and disease control rates can be defined as (CR + PR + SD)/(CR + PR + SD + PD) × 100% [22, 23].

### 3.7. Statistical Treatment

The SPSS 26.0 software was used for statistical analysis of the data involved in this study, and the measurement data were verified [24]. After confirming that the data were normally distributed, mean ± standard deviation (‾*x* ± *s*) was used to represent the data differences between groups, and a *t*-test was performed. The statistical data involved were expressed by (*n*, %), and the differences between groups were analyzed by the *x*^2^ test [25]. The prediction and diagnostic value evaluation of NSCLC patients with brain metastasis were completed by the ROC curve, and *P* < 0.05 proved that the differences were statistically significant.

## 4. Results and Analysis

### 4.1. Comparison of Baseline Data

There were no significant statistical differences in gender, age, and disease type (all *P* > 0.05) and significant statistical differences in pathological stages (*P* < 0.05), as shown in Table 1.

### 4.2. The Postoperative Expression of P53 Protein and miR-424 was Compared

The positive expression rate of P53 protein and the relative expression level of miR-424 in the NSCLC BMS group increased significantly than those in the NSCLC BMS group (all *P* < 0.05), as shown in Table 2.

### 4.3. Analysis of the Predictive Value of the P53 Protein Gene for Brain Metastasis in NSCLC Patients

The predictive efficacy of the P53 protein gene in NSCLC patients with BMS was analyzed by the ROC curve, which showed a high area under the ROC curve (AUC = 0.793), a sensitivity of 80.00%, a specificity of 78.50%, and a Youden index of 0.585.  Figure 1 shows the ROC curve of P53 protein gene detection of brain metastases in NSCLC patients.

### 4.4. Comparison of miR-424 Expression in Serum of Patients before and after Drug Resistance

All 82 NSCLC patients selected in this study were treated with EGFR-TKIs. After 3 months, follow-up investigation was conducted on all patients to evaluate the treatment effect, and the relative expression level of miR-424 in serum samples at the time of initial treatment was detected. Among them, there were 14 patients with complete response (CR), 40 patients with partial response (PR), 22 patients with stable disease (SD), and 6 patients with disease progression (PD). The median relative expression of miR-424 in patients with treatment failure, namely the PD group, was 0.702 (0.425–1.203). The median relative expression of miR-424 was 1.097 (0.507–2.362) in patients with objective remission, namely, the CR + PR + SD group. Comparison between groups showed that the relative expression of miR-424 was lower in the PD group (*P* < 0.05).

## 5. Conclusions

In this study, a retrospective analysis is conducted to analyze the predictive value of P53 protein expression in brain metastases in NSCLC and the mechanism of miR-424-reversing platinum resistance in NSCLC. The results showed that the expression of P53 protein and miR-424 was closely related to the prognosis of patients. In addition, the expression of P53 protein has a high predictive value for the occurrence of BMS in patients with non-small-cell lung cancer. This study also has some limitations. Due to the limited number of retrospective studies and cases, this study also needs to expand the scope of the study to further verify the results. In the future work, we will confirm the clinical value of P53 protein and miR-424 expression in non-small-cell lung cancer through a large-sample prospective randomized controlled study.

## Figures and Tables

**Figure 1:** ROC curve of P53 protein gene detection of brain metastases in NSCLC patients.

**Table 1:** Comparison of baseline data.

Indicators	NSCLC brain metastases group (*n* = 34)	NSCLC without metastasis group (*n* = 48)	*t*/*x*^2^	*P*
Gender (*n*, %)			0.455	0.500
Male	18 (52.94)	29 (60.42)		
Female	16 (47.06)	19 (39.58)		
Age (years)	55.74 ± 8.54	56.00 ± 7.24	−0.149	0.882
Disease types (*n*, %)			0.139	0.710
Squamous cell carcinomas	17 (50.00)	22 (45.83)		
Adenocarcinoma	17 (50.00)	26 (54.17)		
Pathological staging (*n*, %)			5.271	<0.001
Phase I	0 (0.00)	26 (54.17)		
Phase II	20 (58.82)	21 (43.75)		
Phase III	14 (41.18)	1 (2.08)		

**Table 2:** Comparison of postoperative expression of P53 protein and miR-424.

Group	Positive expression rate of P53 protein	Relative expression of miR-424
NSCLC brain metastases group (*n* = 34)	27 (79.41)	1.12 ± 0.26
NSCLC without metastasis group (*n* = 48)	11 (22.92)	0.71 ± 0.11
*t*/*x*^2^	25.546	9.778
*P*	<0.001	˂0.001

## Data Availability

The simulation experiment data used to support the findings of this study are available from the corresponding author upon request.
